# Prediction Method of Gestational Diabetes Based on Electronic Medical Record Data

This article has been retracted.

**DOI:** 10.1155/2021/6672072

**Published:** 2021-03-08

**Authors:** Yang Liu, Zhaoxiang Yu, Hua Sun

**Affiliations:** ^1^Department of Endocrine, Affiliated Hospital of Beihua University, Jilin 132012, China; ^2^Department of Anesthesiology, Affiliated Hospital of Beihua University, Jilin 132012, China

## Abstract

At present, the secondary application of electronic medical records is focused on auxiliary medical diagnosis to improve the accuracy of clinical diagnosis. The main research in this article is the prediction method of gestational diabetes based on electronic medical record data. In the original data, the ID number of the medical examiner did not match the medical examination record. In order to ensure the accuracy of the data, this part of the record was removed. First, the preparation stage before building the model is to determine the baseline accuracy of the original data, test the effectiveness of the machine learning algorithm, and then balance the target data set to solve the bias caused by the imbalance between data classes and the illusion of excessive model prediction results. Then, the disease prediction model is constructed by dividing the data set, selecting parameters and algorithms, and visualizing the model. Finally, the effect of predictive model construction is comprehensively judged based on multiple evaluation indicators and control experimental models. In this paper, the RF model can be used to rank the importance of the feature importance of the output feature on the importance of the classification result of the input feature. In order to test the accuracy of regression prediction, the experiment uses absolute mean error and root mean square error to evaluate the accuracy of fasting blood glucose prediction. A logistic regression model is constructed through the training set, and the test set data are brought into the prediction model for prediction. Experimental data show that when the features filtered by WBFS are used, the accuracy, *F*1 value, and AUC value of logistic regression are 0.809, 0.881, and 0.825, respectively, which is an increase of about 12% compared with when the feature is not used. The results show that the electronic medical record data drive can effectively improve the accuracy of predicting gestational diabetes.

## 1. Introduction

With the increasing dissemination and accumulation of medical data, massive real and effective patient information is stored in the electronic medical record system. The causes of diabetic complications are complex and affected by many factors [1]. In medicine, the significance of chronic disease prevention is higher than that of treatment. Therefore, with the help of information technology and intelligent technology, the main influencing factors can be mined from the rich data of electronic medical record for early prediction, which is convenient for accurate treatment, improvement of medical service quality, and reduction of medical cost.

Biologically speaking, glucose can enter the fetal circulation through the placenta, but insulin cannot. When the fetal pancreas secretes insulin normally, it can promote normal growth and fat development. However, if it maintains hyperglycemia and hyperinsulinemia for a long time, once it leaves the maternal environment through childbirth, it may be complicated with neonatal transient hypoglycemia. In the treatment process of patients with chronic diseases, each examination index has the characteristics of large number and complex relationship. The traditional diagnosis and treatment process requires a large number of doctors with strong professional medical knowledge and experience, and it takes a lot of human and material resources to process a large number of indicators including gene data. Therefore, artificial intelligence and other technologies play a very important role in the prediction and diagnosis of diabetes [2].

Electronic medical records play a certain role in promoting the prediction of gestational diabetes. Rayanagoudar believes that women with gestational diabetes are at risk of developing type 2 diabetes, but the individualized risk estimates are unclear. He conducted a meta-analysis to quantify the risk of developing type 2 diabetes in women with GDM. He systematically searched major electronic databases without language restrictions. He separately extracted 2 × 2 tables for dichotomous data, and mean plus SE for continuous data. He uses a random effects model to calculate and summarize the hazard ratio. Although his research has certain theoretical value, the research method lacks precision [3]. Iliodromiti thinks targeted screening, guided by biomarkers, may be feasible. He tried to determine the accuracy of the early prediction of GDM by circulating adiponectin. He synthesizes data on diagnostic accuracy using bivariate mixed effects and layered summary receiver operating characteristics (HSROC) models. He suggests that measuring circulating adiponectin before and early in pregnancy may improve detection rates in women at high risk for GDM. Although his research is relatively accurate, it is not comprehensive enough [4]. Zhang believes that gestational diabetes mellitus (GDM) is a common complication of pregnancy and remains an important public health and clinical issue. He argues that observational studies conducted over the past decade have identified a number of dietary and lifestyle factors associated with the risk of GDM and have demonstrated that the time frames before and during pregnancy may be associated with the development of GDM. Although his research is relatively accurate, it lacks a specific experimental scheme [5]. Xing et al. believes that gestational diabetes (GDM) is a disease that usually occurs in the second to third trimester of pregnancy. Its pathological conditions include hyperglycemia, hyperinsulinemia, and fetal dysplasia. He uses the antioxidant naringin to further enhance the efficacy of hESC-derived PE transplants. He differentiated insulin-secreting PE from hESC and transplanted it into GDM mice. He administered naringenin to mice receiving PE transplantation, and sham-operated mice were used as negative controls to evaluate its effect on reducing the symptoms of GDM. Although the factors considered in his research are more comprehensive, experimental data are lacking [6].

In theory, to integrate learning algorithm in prediction of direction diseases, this paper provides a case study, rich in the field of artificial intelligence in the medical application, to also make up for the inadequacy of existing gestational diabetes forecast model, provide theoretical methods and algorithms for disease diagnosis model tools, enrich and perfect the personalized model explanation, and help and train of thought for disease diagnosis prediction research in China. In this paper, the experimental results obtained from the test set are compared to obtain the best model.

## 2. Electronic Medical Record Data Drive and Prediction of Gestational Diabetes

### 2.1. Electronic Medical Records

When matching patient records, this article uses clustering of patient records to divide them into many parts. Only records in the same part are matched with each other, which greatly reduces the amount of calculation required for comparison. Through clustering and matching, if several matching records are found, these records need to be merged [7]. The support of each drug set sequence cluster is defined as

(1) $$\begin{array}{c} {\text{Support}}_{k}=\frac{\sum_{j}\lambda \left(C\left({\text{DSS}}_{j}\right),E\left(\text{DSS}C_{k}\right)\right)}{N},\;k=1,2,\ldots ,K. \end{array}$$

According to the defined core patient treatment record set Core_*k*_, the support of all drugs in the cluster *C*_*k*_ is defined as

(2) $$\begin{array}{c} {\text{Support}}_{k}\left(d_{g}\right)=\frac{\sum_{{\text{TR}}_{j}\in {\text{Core}}_{k}}\lambda \left(d_{g},{\text{TR}}_{j}\right)}{\left|{\text{Core}}_{k}\right|},\;g=1,2,\ldots ,M. \end{array}$$

The typical drug set in the cluster *C*_*k*_ is defined as

(3) $$\begin{array}{c} {\text{TDS}}_{k}=\left\{d_{g}|{\text{Support}}_{k}\left(d_{g}\right)>\delta_{1}\right\}, \end{array}$$

where *δ*_1_ is the threshold defined in advance.

For the evaluation of typical medication time, the support of selected indicators is defined as

(4) $$\begin{array}{c} {\text{Support}}_{k}\left(I_{f}\right)=\frac{\sum_{{\text{TR}}_{j}\in {\text{Core}}_{k}}\lambda \left(I_{f},\text{PI}\left({\text{TR}}_{j}\right)\right)}{\left|{\text{Core}}_{k}\right|},\;f=1,2,\ldots ,5. \end{array}$$

In order to realize the function of providing decision support for the diagnosis and treatment of a patient, it is very necessary to obtain the patient's data information from the electronic medical record [8]. Taking logit *p* as the dependent variable, and the factors affecting the dependent variable are *x*_1_, *x*_2_, ..., *x*_*k*_, then

(5) $$\begin{array}{c} \ln\frac{p}{1-p}=b_{0}+b_{1}x_{1}+\cdots +b_{k}x_{k}. \end{array}$$

From the above formula, we can get

(6) $$\begin{array}{c} p=\frac{\exp\left(b_{0}+b_{1}x_{1}+\cdots +b_{k}x_{k}\right)}{1+\exp\left(b_{0}+b_{1}x_{1}+\cdots +b_{k}x_{k}\right)}. \end{array}$$

Under normal circumstances, the network mean square error is selected as the error criterion function; namely,

(7) $$\begin{array}{c} E=E_{e}=\frac{1}{N}\sum_{i=1}^{N}{\left(e_{i}\right)}^{2}=\frac{1}{N}\sum_{i=1}^{N}{\left(t_{i}-o_{i}\right)}^{2},\\ \left\{\begin{array}{c} E=VE_{e}+\left(1-V\right)E_{w},\\ E_{w}=\frac{1}{n}\sum_{j=1}^{n}{\left(w_{j}\right)}^{2}, \end{array}\right. \end{array}$$

where *V* is the scale factor and *n* is the total number of bias values and weights.

The calculation formula of the accuracy rate in the two-classification problem is

(8) $$\begin{array}{c} \text{accuracy}=\frac{n+p}{m+n+p+q}. \end{array}$$

The model of logistic regression is as follows:

(9) $$\begin{array}{c} P\left(Y=1|x\right)=\frac{\exp\left(w\cdot x\right)}{1+\exp\left(w\cdot x\right)},\\ P\left(Y=0|x\right)=\frac{1}{1+\exp\left(w\cdot x\right)}. \end{array}$$

The process of data mining starts from receiving and inputting the original data [9], screening important data items, reducing dimension and concentrating data set, noise reduction, and standardizing data and other preprocessing steps, and then carries out multidimensional analysis, pattern recognition, model evaluation, difference significance analysis, and other work on the data to complete the transmission process of the original data from data to information, and then to knowledge [10, 11]. Because the value of *y* can only be 0 and 1, the loss function is constructed as follows:

(10) $$\begin{array}{c} P\left(y|x;\theta \right)={\left(h\theta \left(x\right)\right)}^{y}{\left(1-h\theta \left(x\right)\right)}^{1-y}. \end{array}$$

The expression of the strong learner is

(11) $$\begin{array}{c} f_{t}\left(x\right)=f_{t-1}\left(x\right)+\sum_{j=1}^{J}c_{tj}I\left(x\in R_{tj}\right). \end{array}$$

Compared with GBDT, Xgboost performs a second-order Taylor expansion on the objective function, and its objective function is

(12) $$\begin{array}{c} {\text{Obj}}^{\left(t\right)}=\sum_{i=1}^{n}l\left(y_{i},{\hat{y}}_{i}^{\left(t-1\right)}+f_{t}\left(x_{i}\right)\right)+\Omega \left(f_{t}\right)+\text{constant}. \end{array}$$

### 2.2. Data Drive

The pattern produced each time is not necessarily what we expect. In some cases, the better patterns we get cannot be well generalized on other data sets, and then the phenomenon of overfitting occurs. The methods to overcome overfitting include regular term and cross-validation. If the pattern obtained through data mining does not meet the required standards, the process of data preprocessing, model training, and result evaluation must be carried out again. At the same time, patients also have many questions and needs in assessing their own health status and making medical decisions [12, 13].

With the continuous development of computer technology and network technology, the ability of using various data or knowledge collected under different backgrounds and different devices has been greatly improved, so the ability of applying these data and knowledge to solve medical problems and make medical decisions has also been greatly improved [14]. The presentation of data mining results should follow the principle of easy analysis and understanding, and try to use tables, flow charts, and other means [15]. In addition, the data mining results are not necessarily effective, or in line with the data mining goal setting. We should use certain indicators to screen out valuable results, evaluate their novelty and effectiveness, and make a summary and analysis of the subject goals and tasks. The hospital electronic medical record data are multisource heterogeneous, distributed in different servers and different databases, so the data should be integrated before data prediction, and the data of patients should be integrated into a complete record [16].

### 2.3. Prediction of Gestational Diabetes

It is worth noting that unsaturated or chemically modified phospholipids can be detected as early as the first trimester, and the levels of these phospholipids are always low throughout in pregnancy. In addition, the trajectory of these phospholipids in the third trimester does not seem to be affected by lifestyle changes in pregnant women with GDM. Some of these diseases can be cured in the neonatal period, and some become the root causes of long-term neonatal diseases [17]. Pregnant women should always pay attention to their physical and mental health. During pregnancy, they should carry out appropriate physical activities, pay attention to controlling the weight before pregnancy and the rate of weight gain during pregnancy, adjust their sleep schedule, and improve their sleep quality as much as possible.

For high-risk GDM pregnant women with a history of spontaneous abortion, medical abortion, assisted reproductive technology, family history of diabetes, and obesity before pregnancy, they should pay more attention to their blood sugar levels during pregnancy to avoid the occurrence of GDM. Therefore, when performing statistical analysis and statistical modeling, first perform data cleaning, detect and delete outliers to ensure a noise-free data set, or predict the results. For data sets with less impact, increase the maximum predictive value of the predictive diagnosis model of gestational diabetes [18–20].

In this paper, we first study the impact of different types of features and multiclass feature combination on disease diagnosis methods, then design a feature screening method to evaluate the importance of features, so as to automatically screen the appropriate number of features, and then use depth representation methods such as network embedding to vectorize features, and analyze the relationship between features through similarity measurement method, and it is applied to the classification model for prediction. This method can automatically learn some features based on domain knowledge rather than artificial rules, so it can often achieve better results [21, 22].

For patients, self-management is a kind of health behavior that patients promote and increase their health through their own activities, control and manage their own conditions, reduce the impact of disease causes on their own physiological function, emotion, and interpersonal and social relations, and adhere to effective management of their own conditions for a long time [23]. Therefore, in this regard, we should not only communicate and educate patients, but also urge them to control their diet and exercise, help them make strict self-management plans, strengthen supervision over patients who cannot complete their tasks on time through appointment review, and communicate with their family members at any time to help them establish a good family atmosphere and have family support. Patients will better cooperate with doctors to complete self-management tasks [24].

## 3. Model Prediction Simulation Experiment

### 3.1. Data Collection

The data set in this paper has 1000 samples, 83 features and complex data structure, including 23 continuous features and 60 discrete features. The number and proportion of missing features are shown in Table 1. In the data set of this paper, almost all the initial diagnosis is consistent with the final diagnosis, which means that the patient's real disease can be identified through the initial diagnosis, but this situation is not realistic in clinic. At the same time, considering the error and nonstandard of information input, this paper will not use the initial diagnosis as a feature to introduce into the constructed classification model [25, 26].

### 3.2. Data Preprocessing

In the original data, the ID number of the medical examiner did not match the medical examination record. In order to ensure the accuracy of the data, this part of the record was removed. For records containing a large number of default values, in order to ensure data quality, these records are also deleted. For the assignment of mass spectral features, the highest score of metabolite candidate is preferred [27].

### 3.3. Model Construction

After preprocessing, such as integration and cleaning, filling and dimensionality reduction, the data can be analyzed. After dimensionality reduction, four data set samples are formed, namely, the non-dimensionality reduction data set and the data set processed by three-dimensionality reduction methods. Firstly, in the preparation stage before the model is constructed, the baseline accuracy of the original data is determined, the effectiveness of the machine learning algorithm is tested, and then the target data set is balanced, so as to solve the bias caused by the imbalance between data classes and the false appearance that the prediction result of the model is too high [28]. Then, the disease prediction model is constructed by dividing data sets, selecting parameters, and selecting algorithms, and the model is visualized. Finally, according to a variety of evaluation indexes and control experimental model, the construction effect of prediction model was comprehensively judged. The ultimate goal is to find the undiscovered but actual domain knowledge, and to realize the formal description of hidden knowledge and transform it into explicit knowledge. In the process of model construction, the overall effect of a model is judged through the 10-fold cross of training set, and then the model is tested according to the most appropriate parameters, because if the parameters of the test set are adjusted, it is easy to over fit, and the model is only suitable for the data set; that is, the generalization ability of the model is not strong [29].

### 3.4. Feature Analysis

In the study of predictive diagnosis of gestational diabetes mellitus, the feature selection of data plays a very important role in the prediction accuracy. In the case of less samples and more features, if the features can be analyzed correctly and the noise can be eliminated, the overall performance and stability of the model can be qualitatively improved [30]. In this paper, the RF model is used to rank the importance of the output features and the influence of the input features on the classification results. According to the relationship between the feature and the sample being generally 1 : 30, and the general IV value is less than 0.05, the feature is removed. Observe the top 40 features; their IV are greater than 0.05, so select the top 40 features to enter the model training [31, 32].

### 3.5. Model Evaluation

According to the generated model, the predicted value of fasting blood glucose in the next year can be obtained by inputting the test set. The predicted value of fasting blood glucose in the third year was subtracted from the predicted value of fasting blood glucose, and the difference was the predicted value of fasting blood glucose change. The difference value indicates the predictive score of fasting blood glucose change, and the difference value with larger absolute value indicates larger change. So far, the prediction of fasting blood glucose in the next year has been transformed into a binary problem. In order to test the accuracy of regression prediction, absolute mean error and root mean square error were used to evaluate the accuracy of fasting blood glucose prediction. The logistic regression model was constructed through the training set, and the test set data was brought into the prediction model for prediction [33].

## 4. Prediction Results of Gestational Diabetes

### 4.1. Comparative Analysis of FPG Levels in Different Periods of Pregnancy

The classification results of EMR data set are shown in Table 2. Compared with the experimental results of CNN model, the diagnostic accuracy and *F*-value of SDG-CNN model on the four EMR data sets are significantly increased, which indicates that integrating medical vocabulary semantics into deep learning model and using prior knowledge to guide model training achieve the purpose of effective use of prior knowledge, so that the model can understand lexical semantic information to a certain extent [34], not just statistical information.

The comparison of insulin-related indicators is shown in Figure 1. Due to the limited retention of serum samples, the consumption of different detection indicators, and the difference of detection reagents between batches, 128 samples were tested for fins, and the correlation between 25(OH)D and insulin was analyzed, including 15 cases in GDM group and 113 cases in normal group. The concentrations of FPG, 25(OH)D, and fins were 4.6 ± 0.4 mmol/L, 28.0 ± 9.4 ng/ml, and 9.9 ± 2.9 mU/L, respectively. HOMA-*β* and HOMA-IR were calculated by the formula and analyzed after natural logarithm transformation.

Figure 2 shows the comparison of FPG value between early pregnancy and OGTT. The FPG values in the early pregnancy and the FPG values in OGTT were compared between the two groups. The results showed that the FPG values in the early pregnancy and OGTT of the GDM group were 5.18 mmol/L and 5.21 mmol/L, respectively, higher than the 4.85 mmo1/L and 4.64 mmol/L of the normal group, and the difference was statistically significant (*p* < 0.05). In the normal group, the FPG value in the early pregnancy was compared with the FPG value at OGTT, and the difference was statistically significant (*p* < 0.05); the GDM group was compared with the FPG value in the early pregnancy and the FPG value at OGTT, and the difference was not statistically significant (*p* < 0.05).

The ROC curve of the modeling model is shown in Figure 3. The GDM risk prediction model for pregnant women in the training modeling population has an AUC of 0.743, a sensitivity of 0.826, a specificity of 0.757, a positive predictive value of 0.585, a negative predictive value of 0.821, and an accuracy of 0.802.

The comparison between GA tuning and grid search tuning results is shown in Table 3. The genetic algorithm used in this paper to find the optimal parameters of CatBoost has the highest *F*1 value and AUC value, which are 0.775 and 0.847, respectively. The cascaded GA-CatBoost gestational diabetes predictive diagnosis model proposed in this paper has an *F*1 value of 0.790 and an AUC value of 0.872 on the test data set.

### 4.2. Algorithm Performance Analysis

The performance comparison of each classifier model is shown in Figure 4. The experimental results show that the cascade GA-Catboost proposed in this paper is superior to support vector machine, artificial neural network, and other ensemble learning algorithms in *F*1 value and AUC value and has good stability and generalization ability. Therefore, the Catboost model optimized by genetic algorithm is selected as the best model for predicting and diagnosing gestational diabetes mellitus [35]. When using the features screened by WBFS, the accuracy, *F*1 value, and AUC value of logistic regression are 0.809, 0.881, and 0.825, respectively, which are about 12 percentage points higher than those without feature screening, reflecting the improvement of WBFS method on the performance of the model.

The model information of GDM data set is shown in Table 4. It can be seen from the table that using stacking model can achieve the best effect. Compared with the baseline accuracy of 0.63, the accuracy of stacking model can reach 0.857. After comparative analysis, it can be found that, when using the network embedding model, the best effect can be achieved by constructing the network topology model of traditional Chinese medicine, choosing the maximum value mapping method, taking the cos similarity as the similarity measure, with the vector dimension of 32 and the threshold value of 0.4, which can improve the accuracy of the classification model by 8 percentage points. This is because, after feature screening, not all features are used, but only some features with high importance are used. In this part of features, the number of TCM features is not very large, which means that the influence of feature learning based on TCM domain knowledge is limited, so only for these features, the improvement of the model is certainly limited.

The change of life style, especially in late pregnancy, is related to the persistence of exercise. Health education activities can improve the patient's awareness of the disease, which is conducive to the change of the patient's activity mode and behavior. After learning the common sense about the disease, the patient will have a new attitude change on how to carry out self-behavior management. The understanding of disease includes the content of health education and the understanding of outcome. The principal component analysis is shown in Table 5. According to the factor load matrix, the eigenvalues of each factor are obtained. There are 8 factors with eigenvalues greater than 1. The size of the first to the eighth principal component characteristic root was 2.743, 2.563, 2.339, 2.190, 1.826, 1.738, 1.507, and 1.119, respectively. The contribution rates of principal components were 10.158%, 9.492%, 8.664%, 8.113%, 6.763%, 6.434%, 5.580%, and 4.144%, respectively. The characteristic root of the ninth attribute is 0.994, accounting for 3.683% of the total contribution rate. The characteristic root of the latter attribute is smaller and smaller, and its contribution to the overall characteristics of the data set is also less and less. Therefore, there are eight principal components in the original variable.

Compare the performance on the random forest of the original data set, the data set with the cross-item added, and the data set after the cross-feature selection. By comparing the value of AUC, the performance of the model is evaluated. The AUC value of the random forest on the original data set and the data set with the cross term is shown in Figure 5. Through comparison, it is found that, after adding the cross term, the model performance has improved, indicating that the cross term contains potential information and can improve the model performance. In the feature selection method, selecting the features that have a strong influence on the model performance from the cross features can effectively improve the model performance. Finally, 227 cross-term features are selected and added.

### 4.3. Model Prediction Results

When the sample size of the test set changes from 10% to 50%, the area under the ROC curve of the three models changes as shown in Figure 6. It can be seen from the figure that the area under the ROC curve of the three models changes little with the change of the sample size of the test set, indicating that the three models have good stability and generalization ability. The area under the ROC curve of BP neural network is larger than that of logistic regression model under the five proportional test sets, which indicates that the prediction accuracy of BP neural network is better than that of traditional logistic regression model. Compared with the traditional statistical model, the neural network model has better prediction performance in predicting the results of multivariable interaction, which may be due to the fact that the neural network model is not affected by the complex interaction between variables and has stronger fitting ability for complex data [36]. Taking blood glucose as independent variable and GA as dependent variable, multiple linear regression analysis and multiple stepwise regression were performed. In GDM, fasting blood glucose was the significant influencing factor of glycosylated albumin; in ODM, fasting blood glucose and OGTT 120 were the significant influencing factors of glycosylated albumin. Multiple stepwise regression analysis of significant variables confirmed that blood glucose had significant effect on GA.

The comparison of clustering results under different similarity measurement methods is shown in Figure 7. For data set 1, when *K* is 2, the maximum stable value is 0.37; when *K* is 3, 4, or 6, the maximum stable value is 0.0286. Similarly, for data set 2, the maximum stability value when *K* is 2 is 0.429, and the maximum stability value when *K* is 3 is 0.143. For data set 3, the maximum stability value when *K* is 2 is 0.235, and when *K* is 3 or 6, the maximum stability value is 0.059. The ROC curve for diagnosing hyperglycemia in pregnancy was drawn with the glycated albumin value. The AUC was 0.89, the diagnostic cut-off value was 12.29%, and the binary logistic regression analysis showed an OR value of 4.271. It can be seen that elevated glycated albumin is abnormal glucose metabolism during pregnancy. The risk factors of the disease have certain diagnostic value. Glycated albumin, as an indicator reflecting the average blood glucose level during pregnancy, is not affected by special physiological changes during pregnancy, and it has important value in predicting the risk of near and long-term complications of the mother and baby.

For pregnant women who developed GDM in the later stage, the content of these phospholipids did not decrease from the first trimester to the second trimester, but overall, there was a slight increase trend from the first trimester to the third trimester. Therefore, most of the selected phospholipid metabolites usually only show significant differences in the early and third trimesters between the two groups. In many cases, metabolites in the second trimester were not statistically different between the two groups, which is consistent with the results of multivariate statistical analysis. The generation time of association rules is shown in Table 6 and Figure 8. It can be seen from the table that the calculation time is basically 5–9 seconds. In general, under the premise of nearly 3 million rows of data, the calculation time is within 10 seconds.

## 5. Conclusions

In the field of medical research, medical record data mining has great research potential. Medical record data mining can provide data support and diagnostic help for medical diagnosis. From the perspective of medical researchers, medical record data mining technology can contribute to its scientific research. The basic information, diagnosis information, and treatment information of patients will be recorded in the electronic medical record system. Through the establishment of electronic medical record system, hospital management can reflect the characteristics of informatization, and patients can enjoy higher quality service.

Hospital data mining technology will be widely used in the hospital information system and is an important technology component of medical information on this specific case. This simple and feasible method is suitable for medical personnel. Through data mining technology, doctors can conduct in-depth exploration and research on the characteristics and laws of diseases, which has great practical value. Monitoring of blood lipid level in early pregnancy can predict gestational diabetes in early stage, and early intervention has important clinical significance for reducing pregnancy complications and avoiding adverse pregnancy outcomes.

In feature selection, the feature importance sequence can be obtained by synthesizing the weight-based feature selection method used in this paper. However, if the weight can be adjusted by combining the domain knowledge of experts, the selected features will be more in line with the actual needs. According to the principle of game theory, the influence of each feature on the prediction model under a posteriori probability is calculated, so as to measure the contribution of the feature. For any sample, the existence of the feature will change the prediction value in the model of the sample, the change caused by the important feature is larger, and the change caused by the secondary feature is smaller.

## Figures and Tables

**Figure 1:** Comparison of insulin-related indicators.

**Figure 2:** Comparison of FPG value in early pregnancy and OGTT.

**Figure 3:** Modeling model ROC curve.

**Figure 4:** Performance comparison of each classifier model.

**Figure 5:** AUC value.

**Figure 6:** Changes in the area under the ROC curve of different models.

**Figure 7:** Comparison of clustering results under different similarity measurement methods.

**Figure 8:** Association rule generation time.

**Table 1:** Feature missing number and missing proportion statistics.

Feature name	Missing number	Missing ratio
SNP22	540	0.54
SNP21	539	0.54
SNP23	538	0.54
SNP55	517	0.52
SNP54	517	0.52
ACEID	517	0.52

**Table 2:** Classification results of EMR data set.

Model	Combination method	Precision (%)	Accuracy (%)	*F*1-score (%)
CNN	pre_pre	83.79	83.49	83.58
	pre_post	83.79	83.55	83.62
	post_pre	83.94	83.72	83.78
	post_post	83.81	83.48	83.58

SDG-CNN	pre_pre	85.87	85.65	85.71
	pre_post	85.82	85.52	85.58
	post_pre	85.92	85.74	85.78
	post_post	85.7	85.47	85.51

**Table 3:** Comparison of GA tuning and grid search tuning results.

	GA-CatBoost	GS-Catboost
*F*1	0.775	0.736
AUC	0.847	0.819

**Table 4:** Model information of the gestational diabetes data set.

	Logistic	SVM	GBDT	Adaboost	XGboost	RF	Extra	Stacking
AUC	0.862	0.86	0.808	0.786	0.739	0.725	0.795	0.922
ACC	0.779	0.786	0.679	0.693	0.643	0.65	0.714	0.857
*F*1	0.768	0.764	0.653	0.668	0.604	0.622	0.692	0.875

**Table 5:** Principal component statistical analysis.

Component	Total	Variance	Cumulative
1	2.743	10.158	10.158
2	2.563	9.492	19.650
3	2.339	8.664	28.31
4	2.190	8.113	36.427
5	1.826	6.763	43.191
6	1.738	6.436	49.627
7	1.507	5.580	55.207
8	1.119	4.144	59.350

**Table 6:** Association rule generation time.

Minconf (%)	20	30	40	50	60	70	20
20	6.51	5.71	5.47	7.30	6.33	7.86	6.51
30	7.44	5.36	5.55	5.48	6.98	6.52	7.44
40	6.41	7.26	7.22	7.27	7.73	7.0	6.41
50	6.36	7.34	5.47	5.75	7.64	8.09	6.36
60	6.93	6.56	5.45	5.56	5.78	8.1	6.93
70	7.67	5.53	5.86	7.45	7.44	7.38	7.67
80	5.55	5.96	6.31	5.91	7.16	5.95	5.55
90	5.75	7.34	5.47	5.86	7.84	5.48	5.75

## Data Availability

No data were used to support this study.
